The article "Clinical Value and Treatment Progress of Prenatal Ultrasonography in Twin Pregnancy: A Systematic Review" was published in 2022. Journal: Contrast Media Mol Imaging.

# Clinical Value and Treatment Progress of Prenatal Ultrasonography in Twin Pregnancy: A Systematic Review

**DOI:** 10.1155/2022/6748487

**Published:** 2022-08-22

**Authors:** Lihua Zou, Jianzheng Yang, Aiping Min, Yang Yin, Minxing Li

**Affiliations:** ^1^Department of Ultrasound, Affiliated Hospital of Southwest Medical University, Luzhou 646000, China; ^2^Department of Ultrasound, City Central Maternal and Child Health Hospital, Leshan 614000, China; ^3^Department of Gynecology and Obstetrics, People's Hospital of Leshan, Leshan 614000, China; ^4^Department of Radiology, People's Hospital of Leshan, Leshan 614000, China

## Abstract

Assisted reproductive technology has continued to develop in recent years, the technology has become more and more mature, and it has improved the total gestational age of the population. Assisted reproductive technology has improved twin pregnancy rates with the use of ovulation-inducing drugs. The risk factor of twins is much higher than singletons, and adverse pregnancy outcomes such as stillbirth and premature birth are more likely to occur than singletons, especially the special complications of monochorionic twins (MC), and the neonatal mortality and morbidity are also increased. Prenatal diagnosis and prognosis of twin pregnancy, as well as therapeutic interventions, are of current concern. Ultrasound can realize the understanding of intrauterine growth and development of twin pregnancy fetuses during pregnancy, can more accurately determine gestational age, organ function, and maturity, and timely detect fetal growth and development abnormalities in twin pregnancy, while the prognosis and treatment still need further improvement. The purpose of this study was to investigate the clinical value and treatment progress of prenatal ultrasound monitoring in twin pregnancy.

## 1. Introduction

With the delay of childbearing age and the increase of elderly pregnant women, especially in the context of the opening of the two-child policy and the widespread development of assisted reproductive technology, the incidence of twin and multiple pregnancy is increasing year-by-year [1]. The birth rate of twin pregnancies increased by nearly 70% from 19% in 1980 to 32% in 2006 [2]. Assisted reproductive technology has continued to develop in recent years, the technology has become more and more mature, and it has improved the total gestational age of the population. Assisted reproductive technology has improved twin pregnancy rates with the use of ovulation-inducing drugs. Twin and multiple pregnancies have become one of the high-risk factors for perinatal morbidity and mortality [3]. Twin pregnancy is a high-risk pregnancy that poses a certain threat to the health of both the mother and the newborn [4]. Compared with singleton pregnancy, the incidence of pregnancy complications caused by twin pregnancy is higher; therefore, prenatal screening of twin pregnancy cannot be ignored [5]. With the continuous advancement of medical imaging technology, ultrasound technology has been further developed and has been widely adopted in prenatal examination of intrauterine fetuses in twin pregnancy [6]. It is one of the most widely adopted, most effective, and easiest methods in obstetrics. This study is a systematic review on the clinical value and treatment progress of prenatal ultrasound monitoring in twin pregnancy.

The article "Clinical Value and Treatment Progress of Prenatal Ultrasonography in Twin Pregnancy: A Systematic Review" was published in 2022. Journal: Contrast Media Mol Imaging.

## 2. Current Status of Prenatal Ultrasonography in Twin Pregnancy

Currently, prenatal diagnosis and prognosis of twin pregnancies, as well as therapeutic interventions, are of great concern. For twin pregnancy, ultrasound plays a prominent role in the monitoring of the whole pregnancy. It is the only means to assess the size of the fetus during pregnancy. It can realize the intrauterine growth and development of the twin pregnancy during pregnancy and can more accurately determine the gestational age. Visceral has an irreplaceable position in the diagnosis and treatment process to detect abnormal fetal growth and development in twin pregnancy in time [7].

In addition to determining the site of pregnancy, judging gestational age, and excluding pathological pregnancy, ultrasonography in early pregnancy can also determine the number of fetuses, the chorionicity of multiple pregnancy, and complications. It is very valuable information for diagnosing fetal growth imbalance, lays an anatomical basis for future selection of intrauterine monitoring methods and intervals, and has a positive significance for reducing perinatal deaths. There are relatively many complications in twin pregnancy, and its prognosis and treatment are still issues that need attention in clinical work. In order to obtain a satisfactory outcome of twin pregnancy, more effective measures are still needed in clinical practice.

## 3. Prenatal Ultrasound Screening and Prevention of Complications in Twin Pregnancy

### 3.1. The Occurrence of Complications in Twin Pregnancy Is Closely Related to Chorionicity

The incidence of twin pregnancies is 1-2%, and the ratio of dichorionic to MC is 3 : 1. Due to the specificity of MC, the pregnancy loss rate in the first and second trimesters is higher compared to dichorionic twins (DC). Therefore, in the routine examination of twins, accurate judgment of chorionicity can help to find twins in high-risk pregnancy, and close inspection and observation can be carried out, and measures can be taken if necessary. MC has higher prenatal and perinatal morbidity than DC [8]. Since twins share the placenta, during the process of placenta formation, blood vessels between the twins form to communicate with each other [9]. When the blood flow on the placenta is unbalanced, complications such as twin-twin transfusion syndrome, intrauterine selective growth restriction, twin reverse arterial perfusion syndrome, and conjoined twins are prone to occur [10]. Therefore, accurate diagnosis of choriopathies during pregnancy has very important guiding significance for clinical practice.

The article "Clinical Value and Treatment Progress of Prenatal Ultrasonography in Twin Pregnancy: A Systematic Review" was published in 2022. Journal: Contrast Media Mol Imaging.

Ultrasound examination is the most important means of monitoring and managing the growth status of twins [11]. It should be closely monitored and the frequency of ultrasonography should be increased if necessary. Transvaginal ultrasound was enrolled at 6–10 weeks of gestation to observe the number of intrauterine gestational sac, germ sac, and yolk sac [12]. The number of gestational sacs is equal to the number of chorions. The early amniotic membrane is not easy to observe, and the yolk sac shows earlier and more clearly than the amniotic sac, so the number of amniotic sacs can be judged according to the number of yolk sacs [13]. However, some scholars put forward a different view that the number of yolk sacs does not represent the number of amniotic sacs, showing a yolk sac twins should continue to follow up until the diagnosis of single amniotic sac [14]. Another reliable evidence is the use of pulse wave and color flow doppler to see umbilical cord entanglement, which is common in monochorionic monoamniotic twin pregnancies, but it is not suitable for early ultrasound diagnosis considering safety issues [15]. From 11–14 weeks of gestation, volume probe reexamination was enrolled for further clarification. Observe whether the amniotic membrane is separated between twins and the shape of the junction with the placenta, whether it is a “T” shaped or a “twin peak” (or “X” sign), the former is MC, which are DC. It has also been reported in the past that the second and third trimesters can be judged according to the sex of the two fetuses, the number of placentas, and the thickness of the diaphragm. However, a large number of practices have proved that the accuracy and sensitivity of judging the chorionicity of twins in the second trimester are lower than that in the early pregnancy. Ultrasound comparison was performed for confirmation. If chorionicity cannot be diagnosed regardless of the evidence, it is recommended that clinical consultation and treatment should be carried out according to MC [16].

### 3.2. Risk Screening and Prevention of Premature Birth in Twin Pregnancy

The rates of spontaneous and iatrogenic preterm births in twin pregnancies are significantly higher than those in singleton pregnancies, especially MC with comorbidities. About 60% of twin pregnancies were delivered prematurely before 37 weeks of gestation and 10% of twin pregnancies were delivered prematurely before 32 weeks of gestation, 5.4 times and 7.6 times that of singleton pregnancies, respectively [17]. The preterm birth prediction method is the same as that of singleton pregnancy, mainly including the medical history, determination of cervical length, and fetal FFN. It is recommended to use transvaginal ultrasound measurement, which has been proved to be a safe, reliable, and repeatable measurement method [18]. Most studies have indicated that a cervical length of less than 25 mm between 18 and 24 weeks of gestation is the cutoff value for predicting preterm birth [19]. Some scholars also believe that in asymptomatic twin pregnancy, when the gestational age is less than 18 weeks, the cervical length less than 30 mm has the highest predictive value for preterm birth before 28 weeks, and the cervical length measurement after the gestational week greater than 22 weeks is more valuable than 28–28 weeks. Preterm birth at 36 weeks had the highest predictive value. Therefore, cervical length measurement is recommended for twin pregnancies before 18 weeks. In addition, in the population of pregnant women with symptoms of preterm birth, the accuracy of predicting preterm birth by cervical length is low [20–23].

The article "Clinical Value and Treatment Progress of Prenatal Ultrasonography in Twin Pregnancy: A Systematic Review" was published in 2022. Journal: Contrast Media Mol Imaging.

There is currently no effective way to prevent premature birth in twin pregnancies. Methods such as bed rest, progesterone therapy, cervical pessary, or oral tocolytics do not reduce the risk of preterm birth in these pregnant women; however, progestin therapy may reduce the risk of neonatal mortality and morbidity [24]. There is no evidence that cervical cerclage, which is well practiced in singleton pregnancy, can prevent the occurrence of premature birth in twin pregnancy. However, most of the current studies on cervical cerclage in twin pregnancy are small sample studies, suggesting that it is urgent cerclage which may reduce the incidence of preterm birth in twin pregnancy and enhance the neonatal survival rate, which needs to be supported by randomized controlled studies with big data [25].

### 3.3. Risk Screening and Prevention of Twin-to-Twin Transfusion Syndrome

The classic ultrasound findings of twin-to-twin transfer syndrome (TTTSA) are as follows: the maximum thickness of the amniotic fluid of the donor child is less than 2 cm, and the maximum diameter of the amniotic fluid of the recipient child is greater than 8 cm; the bladder of the donor child is small or even not full, while the recipient child has a large bladder; occurs in monozygotic twins; the fetal membranes overlap and the placenta lacks arterial-arterial anastomosis [26]; and if the placenta belongs to the donor part, the performance is thin and the echo is strong, while the placenta belongs to the recipient part, the performance is thick and the echo is reduced, and the boundary between the two is often more obvious. Arterial-arterial anastomosis in patients with TTTS has a better prognosis than those who lack it, and arterial-arterial anastomosis seems to prevent the occurrence of TTTS [27].

The article "Clinical Value and Treatment Progress of Prenatal Ultrasonography in Twin Pregnancy: A Systematic Review" was published in 2022. Journal: Contrast Media Mol Imaging.

At present, the treatment options for TTTS include expectant therapy, amniotic fluid reduction surgery, amniotic septostomy, fetoscopic laser coagulation of the communicating branches of the placenta, selective tire reduction, and termination of pregnancy. The best treatment for the diagnosis of TTTS before 26 weeks of pregnancy is fetoscopic laser ablation, and there is evidence that laser ablation has better pregnancy outcomes than amniotic fluid reduction and amniotomy [28]. Some scholars believe that Quintero' I stage should be treated conservatively. Fetoscopic laser ablation was not performed, and amniotic fluid reduction after 26 weeks of gestation was an option. Regardless of early diagnosis (before 16 weeks of gestation) or later diagnosis (after 26 weeks of gestation), laser coagulation is still the best form of treatment for TTTS, and TTTS with a stage higher than stage III has a poor prognosis, with a perinatal fetal loss rate of 70–100%, especially those less than 26 weeks of pregnancy [29]. The amniotic fluid reduction surgery amniotic septostomy, because the operation will increase the risk of premature fetal birth and other risks, is currently and rarely used. However, neurological dysfunction is a serious long-term complication of TTTS regardless of whether treatment measures are taken. In pregnancies with TTTS, the incidence of neurological abnormalities after laser coagulation was 5%, serial amniotic fluid reduction was 14%, and expectant treatment was 21% [30].

### 3.4. Risk Screening and Prevention of Selective Fetal Growth Restriction (SFGR)

SFGR is another common complication of twin pregnancy, with an incidence of about 10–15%. Different countries have different diagnostic criteria for SFGR. Currently, the consensus is that one of the twins has an estimated body mass less than the 10th percentile of the corresponding gestational age and the difference between the twins is greater than 25% [31, 32]. Differences in body mass greater than 20% suggest adverse pregnancy outcomes. The formula is (weight of larger fetus−weight of smaller fetus)/weight of larger fetus. Estimates of fetal weight are primarily derived from ultrasound measurements combined with measurements of the head, abdomen, and femur [33]. SFGR is classified according to the performance of umbilical artery end-diastolic blood flow [34]. Type I has lack of end-diastolic blood flow and reverse umbilical artery; Doppler waveform has positive end-diastolic blood flow, and the survival rate is greater than 90%. Type II has persistent absence and reversal of end-diastolic blood flow: high risk of intrauterine stillbirth in one twin, delayed neurodevelopment of the surviving fetus, and high incidence of preterm birth. The absence and reverse of intermittent end-diastolic blood flow in m-type SFGR leads to unpredictable sudden death in 10–20% of small fetuses and neurological sequelae in 20% of large fetuses.

The article "Clinical Value and Treatment Progress of Prenatal Ultrasonography in Twin Pregnancy: A Systematic Review" was published in 2022. Journal: Contrast Media Mol Imaging.

There are not many reports on the application of SFGR in MC, so there is a lack of high-level evidence to support the application value of SFGR. The intervention plan for twin pregnancy is mainly conservative treatment. In addition, according to the specific conditions of the pregnant woman and the fetus, early termination of pregnancy, laser ablation, and fetal reduction can also be selected. For type I SFGR, the treatment plan is mainly expectant treatment and timely termination of pregnancy. For type II and type *m* SFGR, factors such as the severity of the disease, gestational age, the patient's willingness, surgical risk, and the operator's experience and skills should be considered comprehensively [35].

### 3.5. Risk Screening and Prevention and Treatment of Twin Anemia

Twin anemia-polycythemia sequence (TAPS) has been rarely reported before, and its natural history and effects on fetuses and neonates are still under study. The natural incidence rate is as high as 5%, which often occurs after 30 weeks of gestation, and the probability of TAPS after secondary TTTS laser ablation is as high as 13% [36]. At present, it is believed that the pathogenesis is that there are a small number of small one-way arterial-venous anastomosis vessels in the two fetuses, and there are no compensatory arterial-arterial anastomosis vessels, resulting in chronic low-velocity blood transfusion. However, the clinical manifestations are diverse, which is the gold standard for diagnosis. In addition, the placental echo and thickness are different. The echo of the placenta of the donor fetus is enhanced and the thickness is increased, while the placenta of the recipient fetus has a thinner weak echo area. Due to the decrease in the echo of the liver parenchyma and the increase in the brightness of the portal vein wall, the “starry sky” sign appears in the liver of the fetus with polycythemia. With the aggravation of the disease, the blood-supplying fetus may appear due to cardiac enlargement and edema [37, 38]. Different severity of TAPS may lead to different pregnancy outcomes in twin pregnancies. Severe TAPS can have serious effects on the fetus, and it can cause intrauterine death in twins. The effects of mild TAPS on the fetus are manageable, and twins with this condition may still be born healthy (unless there is a significant difference in hemoglobin levels).

The article "Clinical Value and Treatment Progress of Prenatal Ultrasonography in Twin Pregnancy: A Systematic Review" was published in 2022. Journal: Contrast Media Mol Imaging.

Experience in the treatment of TAPS is also very limited, and management should be individualized. Common methods include conservative management, early delivery, laser ablation of the donor fetus and intrauterine blood transfusion (IUT), combined donor fetal IUT, and donor fetal exchange. Fetal ultrasound monitoring after TTTS fetoscopic laser ablation is particularly important, mainly to monitor the MCA-PSV of twins, and improved fetoscopic laser ablation is the best method to prevent the occurrence of TAPS [39].

### 3.6. Risk Screening and Prevention of Reverse Arterial Perfusion Sequence Syndrome in Twins

Twin reverse arterial perfusion (TRAP) sequence sign, also known as acardiac malformation sequence sign, is characterized by the presence of signs of reverse arterial blood supply or obvious acardiac malformation mass supplied by normal fetal perfusion. Fetal transfusion syndrome, if not diagnosed and treated in time, can lead to high-output heart failure, polyhydramnios, and even intrauterine stillbirth in pumping infants. The prognostic factors of blood pumping infants are complex and are related to the fetal structure, growth and development speed and blood flow, the structure of blood pumping infants, the function of the heart and brain, the nature of amniotic membrane between twins, the umbilical cord, and the volume of amniotic fluid.

If the fetal blood flow is naturally blocked without cardiac malformation in the natural course of the embryo, and early ultrasound diagnosis and timely use of vascular coagulation technology to reduce the fetus, there will be a good prognosis [40].

## 4. New Technology and Development of Prenatal Ultrasound Diagnosis of Twins

### 4.1. Development of Three-Dimensional Ultrasonography and Its Application in Prenatal Diagnosis of Twins

Prenatal 3D ultrasound imaging technology has developed rapidly in recent years, and this technology relies on the advancement of computer technology and image processing technology. Compared with traditional 2D ultrasound imaging, the application of 3D ultrasound imaging in obstetrics has obvious advantages. Advantages are as follows: (1) standardization of ultrasound scanning: two-dimensional ultrasound obtains a cross-sectional image of the fetus, while three-dimensional ultrasound obtains its stereoscopic ultrasound image database by scanning the region of interest, so that ultrasound scanning can be programmed and standardized; (2) intuitive image display: 3D ultrasound can directly display the three-dimensional structure of the region of interest, and 3D ultrasound provides a variety of display modes: surface imaging can visually display the fetal body surface structure; transparent imaging can clearly display the fetal spine and other skeletal structures; (3) overall shape and continuity: multiplane imaging can observe the region of interest from multiple angles and can quickly obtain the plane required for diagnosis. Choose different display modes and the cooperation of various modes according to your needs, which especially provides an important basis for the diagnosis of twins, which helps to enhance the diagnostic information and improve the diagnostic accuracy; (4) accurately locate the diseased tissue: 3D ultrasound imaging can provide doctors with the spatial position and 3D shape of the diseased tissue in the body, thus providing help for intrauterine ultrasound-guided interventional treatment operations; (5) accurate measurement: through 3D reconstruction, it is easier to obtain the standard plane required for measurement, thereby improving the accuracy of measurement of structural parameters such as distance and circumference; more importantly, 3D ultrasound can directly obtain the volume of irregular objects that cannot be measured by 2D ultrasound and use 3D ultrasound to measure fetal vital organs volume, which can effectively evaluate the growth and development status of the fetus; and (6) remote consultation, retrospective analysis of data, and teaching: the stereoscopic image database obtained by 3D ultrasound scanning can provide ultrasound slice maps required for diagnosis and the images have a spatial relationship. After the patient leaves, the doctor can extract the database information for repeated retrospective analysis or through network for remote communication and consultation.

The article "Clinical Value and Treatment Progress of Prenatal Ultrasonography in Twin Pregnancy: A Systematic Review" was published in 2022. Journal: Contrast Media Mol Imaging.

### 4.2. Judgment of Chorionicity in Twins by Three-Dimensional Ultrasonography

Two-dimensional ultrasound indicators are not ideal such as twins with inconsistent sex or two independent placentas can be diagnosed as DC on ultrasound, but it is difficult to determine chorionicity when the sex is the same or the placenta is fused; two-dimensional ultrasound measures the thickness of the septum. The interobserver and intraobserver variabilities in judging chorionicity are large, and it is difficult to accurately diagnose chorionicity by this method in clinical practice [41]. In order to enhance the diagnostic accuracy of twin choriocarcinoma in the second and third trimesters, a combination of multiple ultrasound indicators is currently adopted in clinical diagnosis, but the accuracy is still lower than that in the first trimester. DC has a thicker septum consisting of two layers of amniotic membrane and two chorionic membranes, while MC has a thinner septum consisting of only two amniotic membranes. These histological features contribute to the production of preultrasound, which was used to determine the chorionicity of twins by observing the thickness of the septum. This cutoff value was the most accurate in diagnosing chorionicity regardless of whether two-dimensional or three-dimensional ultrasound was used. Because MC are prone to serious and special complications, the perinatal mortality rate is higher than DC, and clinically, they are more inclined to accept a slightly higher false-positive diagnostic method. Studies have indicated that in the second and third trimesters of pregnancy, the sensitivity, specificity, and accuracy of measuring the thickness of the septum between twins by three-dimensional ultrasonography are higher than two-dimensional ultrasonography, that is, the missed diagnosis rate and misdiagnosis rate of MC are the same. This may be due to the inaccuracy and poor repeatability of the measurement results of the two-dimensional ultrasound on the oblique image of the septal membrane; while, the three-dimensional ultrasound technology reconstructs the three-dimensional image of the septal membrane through the stored volume database, and the septal membrane and the volume of the septum can be observed from different angles and directions. The adjacent relationship provides an opportunity to measure the thickness of the septum vertically, and the most thickness measurement point can be found by rotating the *X*, *Y*, and *Z* axes, so the measurement results are more accurate. In the middle and late pregnancy, H-dimensional ultrasound is adopted to measure the thickness of the septum between twins. The reliability of judging chorionicity is high and repeatability is good. The research results of Seat et al. also show that this method has high accuracy and good repeatability [42]. However, this method is also flawed. This technique is affected by the sample size and gestational age. It still has a certain misdiagnosis rate in judging chorionicity. Therefore, its diagnostic accuracy varies with gestational age and needs to be further studied. This operation method is relatively cumbersome, but easy to learn and can be mastered in a short time. There are several suggestions for operation: select the 3D surface imaging mode and try to make the direction of the sound beam perpendicular to the septum; position the sampling frame on the sagittal plane of the septum to collect 3D volume data; when analyzing the obtained volume data, the transparency adjustment range is set to 20–60, and the minimum threshold adjustment range is set to 10–40. The h-dimensional image of the separation film obtained at this time is more intuitive, vivid, and easy to measure. In addition, by rotating the *X*, *Y*, and *Z* axes, the separation film can be observed from multiple angles and the best measurement position can be found, and then, the measurement vernier can be placed on both sides of the separation film for vertical measurement. It is feasible to use three-dimensional ultrasound to measure the thickness of the septum between twins in the second and third trimesters of pregnancy to determine the chorionicity, and the accuracy and repeatability are good.

The article "Clinical Value and Treatment Progress of Prenatal Ultrasonography in Twin Pregnancy: A Systematic Review" was published in 2022. Journal: Contrast Media Mol Imaging.

### 4.3. Measurement of NT Value in Twins

Ultrasonography is the only method for measuring fetal NT thickness at present. The measurement of NT value in twins is particularly important. Increased NT values are often associated with twin-twin transfusion syndrome, twin-twin arterial reflux syndrome, and twin-twin embolism syndrome. It has two methods: transabdominal ultrasound and transvaginal ultrasound. Since transvaginal ultrasound cannot be accepted by most people during early pregnancy in my country, transabdominal ultrasound is often adopted in China. Two-dimensional ultrasound is routinely adopted for NT measurement during early pregnancy, and three-dimensional volume data are not collected with any slice. During the process, when fetal NT can be clearly observed, only after three-dimensional rotation can the required midsagittal section be obtained, and the NT thickness can be clearly displayed. Meanwhile, the facial structure of the transverse and coronal sections can be displayed through the B and C planes to define whether the three-dimensionally rotated slice is a standard midsagittal slice. Pau et al. believed that three-dimensional ultrasound could be used to measure NT [43]. They believe that it is feasible to use 3D ultrasonic rotation technology to measure NT, and the thickness of NT can be clearly displayed only in 3D acquisition. Ask the examining doctor to have a certain degree of patience to find the standard measurement section. After 3D thermal volume sampling, the 11JI or 3DXI technology of 3D ultrasound can also be adopted for data postprocessing. It can display multiple images on the same plane with a difference of 0.1 mm between each image, which saves relative savings in the process of finding the midsagittal section. Many scholars have been arguing whether 3D ultrasound can be adopted for NT measurement. The early 3D ultrasound instruments had low resolution, and the obtained 3D images were blurry, so accurate measurements could not be performed, and 3D ultrasound can clearly show structures that were not previously visible. This also makes it possible to measure NT using three-dimensional ultrasound.

The article "Clinical Value and Treatment Progress of Prenatal Ultrasonography in Twin Pregnancy: A Systematic Review" was published in 2022. Journal: Contrast Media Mol Imaging.

### 4.4. 3D Contrast-Enhanced Ultrasound

In recent years, three-dimensional contrast-enhanced ultrasound technology has been widely used in the diagnosis of various diseases. This technology has been used in the prenatal diagnosis of twins and has progressed rapidly and achieved good application results. At present, some scholars use this technology, which makes it possible to observe the whole process of arterial perfusion without and reverse in real time. After the contrast agent is injected, the perfusion sequence is exactly the blood perfusion sequence: the umbilical vein of the pumping child ⟶ the body of the pumping child ⟶ the umbilical artery of the pumping child ⟶ the placenta (arterial anastomosis) ⟶ the umbilical artery of the fetus without heart malformation ⟶ the body of the heart malformation ⟶ heartless malformed fetal umbilical vein ⟶ placenta (vein and vein anastomosis) a pumping child umbilical vein. It confirms the characteristics of heartless reverse arterial perfusion circulation, which is consistent with the theory of “arterial perfusion reverse perfusion” generally accepted. It is reported in the literature that there is a remnant heart beat in the chest cavity of acardiac malformation during routine ultrasound examination. Angiography confirmed that the heart remnant has no blood pumping function. Only a little blood flow signal and pulsating blood flow spectrum in the remnant heart can be noticed. By observing the heart rate inconsistent with the vascular pulsation frequency, its blood circulation is still dependent on pumping blood.

Conclusively, ultrasound plays a very important role in the prenatal diagnosis of twins, especially the application of three-dimensional ultrasound, which has opened a new chapter in the prenatal diagnosis of twins, although three-dimensional ultrasound can also form artifacts such as motion, but the three-dimensional or four-dimensional STIC technology has an important application value in the convenience of fetal cardiac ultrasonography. Three-dimensional ultrasonography and STIC technology have their unique advantages and provide more accurate information for prenatal diagnosis of twins, and it is believed that the development prospect is broad.

The article "Clinical Value and Treatment Progress of Prenatal Ultrasonography in Twin Pregnancy: A Systematic Review" was published in 2022. Journal: Contrast Media Mol Imaging.

## Data Availability

The datasets used and analyzed during the current study are available from the corresponding author upon request.

## References

[1] National Collaborating Center for Women’s and Children’s Health (UK) (2011). *Multiple Pregnancy: The Management of Twin and Triplet Pregnancies in the Antenatal Period[M]*.

[2] Hamilton B. E., Martin J. A., Ventura S. J. (2010). Births: preliminary data for 2009[J]. *National Vital Statistics Reports*.

[3] Sebire N. J., Snijders R. J. M., Hughes K., Sepulveda W., Nicolaides K. H. (1997). The hidden mortality of monochorionic twin pregnancies. *BJOG: An International Journal of Obstetrics and Gynaecology*.

[4] Joseph K., Liu S., Liu K. (2003). A parsimonious explanation for intersecting perinatal mortality curves: understanding the effect of plurality and of parity. *BMC Pregnancy and Childbirth*.

[5] Hack K. E. A., Derks J. B., Elias S. G. (2008). Increased perinatal mortality and morbidity in monochorionic versus dichorionic twin pregnancies: clinical implications of a large Dutch cohort study. *BJOG: An International Journal of Obstetrics and Gynaecology*.

[6] Southwest Thames Obstetric Research Collaborative (STORK) (2012). Prospective risk of late stillbirth in monochorionic twins: a regional cohort study. *Ultrasound in Obstetrics and Gynecology*.

[7] Monteagudo A., Roman A. S. (2005). Ultrasound in Multiple gestations: twins and other Multifetal pregnancies. *Clinics in Perinatology*.

[8] Branum A. M., Schoendorf K. C. (2003). The effect of birth weight discordance on twin neonatal mortality. *Obstetrics & Gynecology*.

[9] Harper L. M., Weis M. A., Odibo A. O., Roehl K. A., Macones G. A., Cahill A. G. (2013). Significance of growth discordance in appropriately grown twins. *American Journal of Obstetrics and Gynecology*.

[10] Yinon Y., Mazkereth R., Rosentzweig N., Jarus-Hakak A., Schiff E., Simchen M. J. (2005). Growth restriction as a determinant of outcome in preterm Discordant twins. *Obstetrics & Gynecology*.

[11] Mazher S. B., Kanwal S. (2010). Twin birth weight discordance: associated factors and outcome. *Journal of the College of Physicians and Surgeons Pakistan: JCPSP*.

[12] Appleton C., Pinto L., Centeno M., Clode N., Cardoso C., Graça L. M. (2007). Near term twin pregnancy: clinical relevance of weight discordance at birth. *Journal of Perinatal Medicine*.

[13] Bromley B., Benacerraf B. R. (1995). Using the number of yolk sacs to determine amnionicity in early first trimester monochorionic twins. *Journal of Ultrasound in Medicine*.

[14] Murakoshi T., Ishii K., Matsushita M., Shinno T., Naruse H., Torii Y. (2010). Monochorionic monoamniotic twin pregnancies with two yolk sacs may not be a rare finding: a report of two cases. *Ultrasound in Obstetrics and Gynecology*.

The article "Clinical Value and Treatment Progress of Prenatal Ultrasonography in Twin Pregnancy: A Systematic Review" was published in 2022. Journal: Contrast Media Mol Imaging.

[15] Dias T., Mahsud-Dornan S., Bhide A., Papageorghiou A. T., Thilaganathan B. (2010). Cord entanglement and perinatal outcome in monoamniotic twin pregnancies. *Ultrasound in Obstetrics and Gynecology*.

[16] Guideline Development Group (GDG) members, Ashfaq K. (2011). *NICE Clinical Guideline 129 - the Management of Twin and Triplet Pregnancies in the Antenatal period[J]*.

[17] Martin J. A., Hamilton B. E., Sutton P. D. (2008). Births: Final data for 2006[J]. *National Vital Statistics System*.

[18] Sonek J. D., Iams J. D., Blumenfeld M., Johnson M., Landon S., Gabbe S. (1990). Measurement of cervical length in pregnancy: comparison between vaginal ultrasonography and digital examination. *Obstetrics & Gynecology*.

[19] Yang J. H., Kuhlman K., Daly S., Berghella V. (2000). Prediction of preterm birth by second trimester cervical sonography in twin pregnancies. *Ultrasound in Obstetrics and Gynecology*.

[20] Dai H. (2018). Correlation between the prediction of cervical length measurement and the delivery time of pregnant women with threatened preterm birth[J]. *The Journal of Cardiovascular Surgery: Electronic Edition*.

[21] Sun H. (2019). Predictive value of cervical length detected by perineal ultrasonography in preterm birth in high-risk and threatened preterm women[J]. *China Medical Innovation*.

[22] Conde-Agudelo A., Romero R., Hassan S. S., Yeo L. (2010). Transvaginal sonographic cervical length for the prediction of spontaneous preterm birth in twin pregnancies: a systematic review and metaanalysis[J]. *American Journal of Obstetrics and Gynecology*.

[23] Kindinger L., Poon L., Cacciatore S. (2016). The effect of gestational age and cervical length measurements in the prediction of spontaneous preterm birth in twin pregnancies: an individual patient level meta-analysis. *BJOG: An International Journal of Obstetrics and Gynaecology*.

[24] Romero R., Nicolaides K., Conde-Agudelo A. (2012). Vaginal progesterone in women with an asymptomatic sonographic short cervix in the midtrimester decreases preterm delivery and neonatal morbidity: a systematic review and metaanalysis of individual patient data. *American Journal of Obstetrics and Gynecology*.

[25] Rebarber A., Bender S., Silverstein M., Saltzman D. H., Klauser C. K., Fox N. S. (2014). Outcomes of emergency or physical examination-indicated cerclage in twin pregnancies compared to singleton pregnancies. *European Journal of Obstetrics & Gynecology and Reproductive Biology*.

The article "Clinical Value and Treatment Progress of Prenatal Ultrasonography in Twin Pregnancy: A Systematic Review" was published in 2022. Journal: Contrast Media Mol Imaging.

[26] Kateb A. E., Ville Y. (2008). Update on twin-to-twin transfusion syndrome[J]. *Best Practice & Research Clinical Obstetrics & Gynaecology*.

[27] Taylor M. J. O., Denbow M. L., Tanawattanacharoen S., Gannon P., Cox N., Fisk N. M. (2000). Doppler detection of arterio-arterial anastomoses in monochorionic twins: feasibility and clinical application. *Human Reproduction*.

[28] Roberts D., Neilson J. P., Kilby M. D., Gates S. (2014). Interventions for the treatment of twin-twin transfusion syndrome. *Cochrane Database of Systematic Reviews*.

[29] Simpson L. L. . (2013). Twin-twin transfusion syndrome[J]. *Clinics in Perinatology*.

[30] Quarello E., Molho M., Ville Y. (2007). Incidence, mechanisms, and patterns of fetal cerebral lesions in twin-to-twin transfusion syndrome. *Journal of Maternal-Fetal and Neonatal Medicine*.

[31] Valsky D. V., Eixarch E., Martinez J. M., Crispi E., Gratacós E. (2010). Selective intrauterine growth restriction in monochorionic twins: pathophysiology, diagnostic approach and management dilemmas. *Seminars in Fetal and Neonatal Medicine*.

[32] Sueters M., Oepkes D. (2014). Diagnosis of twin-to-twin transfusion syndrome, selective fetal growth restriction, twin anaemia-polycythaemia sequence, and twin reversed arterial perfusion sequence. *Best Practice & Research Clinical Obstetrics & Gynaecology*.

[33] Stirrup O. T., Khalil A., D’Antonio F., Thilaganathan B. (2015). Fetal growth reference ranges in twin pregnancy: analysis of the Southwest Thames Obstetric Research Collaborative (STORK) multiple pregnancy cohort. *Ultrasound in Obstetrics and Gynecology*.

[34] Gratacós E., Lewi L., Muñoz B. (2007). A classification system for selective intrauterine growth restriction in monochorionic pregnancies according to umbilical artery Doppler flow in the smaller twin. *Ultrasound in Obstetrics and Gynecology*.

[35] Sun L. (2012). Clinical classification, diagnosis and management of selective fetal growth restriction[J]. *Journal of Practical Obstetrics and Gynecology*.

[36] Ville Y. (2006). Prevalence and management of late fetal complications following successful selective laser coagulation of chorionic plate anastomoses in twin-to-twin transfusion syndrome[J]. *American Journal of Obstetrics and Gynecology*.

[37] Slaghekke F., Kist W. J., Oepkes D. (2010). Twin anemia-polycythemia sequence: diagnostic criteria, classification, perinatal Management and outcome. *Fetal Diagnosis and Therapy*.

[38] Lopriore E., Slaghekke F., Oepkes D., Middeldorp J. M., Vandenbussche F. P. H. A., Walther F. J. (2010). Hematological characteristics in neonates with twin anemia-polycythemia sequence (TAPS). *Prenatal Diagnosis*.

[39] Dhillon R. K., Hillman S. C., Pounds R., Morris R. K., Kilby M. D. (2015). Comparison of Solomon technique with selective laser ablation for twin-twin transfusion syndrome: a systematic review. *Ultrasound in Obstetrics and Gynecology*.

The article "Clinical Value and Treatment Progress of Prenatal Ultrasonography in Twin Pregnancy: A Systematic Review" was published in 2022. Journal: Contrast Media Mol Imaging.

[40] Wen Y., Li K., Wang Ke (2015). Perioperative nursing of a case of twin-to-twin transfusion syndrome with fetoscopic laser vascular coagulation[J]. *Chinese Journal of Practical Nursing*.

[41] Stenhouse E., Hardwick C., Maharaj S., Webb T., Kelly F. M., Mackenzie F. M. (2002). Chorionicity determination in twin pregnancies: how accurate are we?. *Ultrasound in Obstetrics and Gynecology*.

[42] Senat M. V., Quarello E., Levaillant J. M., Buonumano A., Boulvain M., Frydman R. (2006). Determining chorionicity in twin gestations: three-dimensional (3D) multiplanar sonographic measurement of intra-amniotic membrane thickness. *Ultrasound in Obstetrics and Gynecology*.

[43] Paul C., Krampl E., Skentou C., Jurkovic D., Nicolaides K. H. (2001). Measurement of fetal nuchal translucency thickness by three-dimensional ultrasound. *Ultrasound in Obstetrics and Gynecology*.

